The article "COVID-19 Risk Prediction for Diabetic Patients Using Fuzzy Inference System and Machine Learning Approaches" was published in 2022. Journal: J Healthc Eng.

# COVID-19 Risk Prediction for Diabetic Patients Using Fuzzy Inference System and Machine Learning Approaches

**DOI:** 10.1155/2022/4096950

**Published:** 2022-04-01

**Authors:** Alok Aggarwal, Madam Chakradar, Manpreet Singh Bhatia, Manoj Kumar, Thompson Stephan, Sachin Kumar Gupta, S. H. Alsamhi, Hatem AL-Dois

**Affiliations:** ^1^School of Computer Science, University of Petroleum & Energy Studies (UPES), Bidholi, Dehradun, India; ^2^Department of Computer Science & Engineering, Amity School of Engineering and Technology, Amity University Uttar Pradesh, Noida, India; ^3^School of Electronics and Communication Engineering, Shri Mata Vaishno Devi University, Katra, India; ^4^Software Research Institute, Athlone Institute of Technology, TUS, Athlone, Ireland; ^5^Department of Electrical Engineering, IBB University, Ibb, Yemen

## Abstract

Individuals with pre-existing diabetes seem to be vulnerable to the COVID-19 due to changes in blood sugar levels and diabetes complications. As observed globally, around 20–50% of individuals affected by coronavirus had diabetes. However, there is no recent finding that diabetic patients are more prone to contract COVID-19 than nondiabetic patients. However, a few recent findings have observed that it could be at least twice as likely to die from complications of diabetes. Considering the multifold mortality rate of COVID-19 in diabetic patients, this study proposes a COVID-19 risk prediction model for diabetic patients using a fuzzy inference system and machine learning approaches. This study aimed to estimate the risk level of COVID-19 in diabetic patients without a medical practitioner's advice for timely action and overcoming the multifold mortality rate of COVID-19 in diabetic patients. The proposed model takes eight input parameters, which were found as the most influential symptoms in diabetic patients. With the help of the various state-of-the-art machine learning techniques, fifteen models were built over the rule base. CatBoost classifier gives the best accuracy, recall, precision, F1 score, and kappa score. After hyper-parameter optimization, CatBoost classifier showed 76% accuracy and improvements in the recall, precision, F1 score, and kappa score, followed by logistic regression and XGBoost with 75.1% and 74.7% accuracy. Stratified k-fold cross-validation is used for validation purposes.

## 1. Introduction

HE development of a novel coronavirus, severe acute respiratory syndrome-coronavirus 2 (SARS-CoV-2), has contributed an unprecedented challenge for the healthcare community around the world. Higher infectivity and comparatively low virulence have caused the rapid transmission of the coronavirus disease 19 (COVID-19) all around the world. Since its earliest instance on December 8, 2019, in the Hubei province of China, COVID-19 has spread into many countries worldwide together with 21,294,845 cumulative cases and 7,61,779 deaths reported globally [1]. COVID-19 symptoms often occur 2 to 14 days after infection, which includes fever (98.6%), cough (59.4%), and sore throat (5%). Many advanced technologies are considered to combat COVID-19 and reduce human interaction [2–5]. Moreover, it is also found in the latest investigations that age, sex, and recent travel history, along with preexisting medical conditions, also played a vital role in the case of COVID-19. It may lead to serious problems [6], such as pneumonia or death. Patients who have diabetes have an elevated risk of serious complications such as adult respiratory distress [7–9]. Though there is no recent finding that people with diabetes are more likely to contract COVID-19 than people with no diabetes, few recent findings observed that it could be at least twice as likely to die from complications of diabetes. Diabetes was shown to be a disease in 22% of the 32 nonsurvivors in a study of 52 trauma patients [10], 16.2% from the study of 173 patients with acute disease, and 12% from the study of 140 hospitalized patients [11, 12]. A twofold gain in the prevalence of patients in intensive care with diabetes has been detected compared with nondiabetic patients concerning COVID-19. Mortality appears to be about threefold greater in people with diabetes [1, 10–13]. Diabetic patients have been observed at greater risk of COVID-19. Few recent studies have demonstrated that the probability of fatal results from COVID-19 is up to 50% greater in patients with diabetes [14].

The machine learning (ML) approach is taken in [15], and a bunch of classification algorithms such as support vector machine (SVM), decision tree (DT), and K-nearest neighbor (KNN) is employed on COVID-19 data. An adaptive neuro-fuzzy inference system (ANFIS) is used to create the dataset for disease risk levels. Over these data, SVM provided 100% accuracy, but when tested against the test data it resulted in 80% risk prediction. Similarly, a bunch of patient data is acquired along with their treatment approaches as categorical values along with the patient's geographical origin and survival count [16]. A random forest approach was taken, and further, this algorithm was boosted by the AdaBoost algorithm, resulting in an impressive 0.86 F1 score. It also gave the probability of survival rate based on the travel history, citizenship, gender, and age group. Kerk et al. [17] established the parametric conditions for the Takagi–Sugeno–Kang fuzzy inference system model to operate as an n-ary aggregation function via fuzzy membership functions and fuzzy rule specifications.

Given the multifold mortality rate of COVID-19 in diabetic patients, this work proposes a COVID-19 risk prediction model for diabetic patients using a fuzzy inference system and machine learning approaches. The proposed model takes eight input parameters, which were found as the most influential symptoms in diabetic patients who contracted COVID-19, namely fever, cough, sore throat, cardiovascular disease, high blood pressure, age, sex, and travel history concerning the last three weeks. Possible five levels of cough, namely chest cough, dry tickling cough, bronchitis, post-viral cough, and whooping cough, have been considered. In the same way, all probable phases of fever are considered. Sex has also played another critical factor in COVID-19. A mean of all significant suffering states recorded 61.8% of cases caused to males, with 38.2% being female. The case fatality rate for COVID-19 is proven to be almost 1.4% gains with age.

Computational intelligence techniques [18–22] such as fuzzy logic are applied to numerous applications [23–25]. A fuzzy logic controller manipulates the linguistic and inexact data, which are not to model the process. In our case, expert knowledge is gained from a few medical practitioners' experiences in treating various diseases such as COVID-19. It can simulate human intelligence and allow the application of real-world rules such as how humans think. Iwendi et al. [16] have used an adaptive neuro-fuzzy inference system (ANFIS) to model and control ill-defined and uncertain systems to predict the risk factors for COVID-19. Classification of COVID-19 dataset has been done using support vector machine, which gave 100% accuracy among all classifiers. Thus, a risk prediction of 80% has been achieved for COVID-19 patients. Furthermore, the authors of [16] used various information related to COVID-19 patients, such as travel, health, and age, to predict the severity of COVID-19. The random forest model has been used for this prediction, which is boosted by the AdaBoost algorithm. As a result, an accuracy of 94% with an F1 score of 0.86 has been achieved. Moreover, the authors of [17] established the parametric conditions for the Takagi–Sugeno–Kang fuzzy inference system model to operate as an n-ary aggregation function via the specifications of fuzzy membership functions and fuzzy rules.

A fuzzy controller can be used to grade uncertainty and imprecision in a certain domain of knowledge. Domain-specific knowledge and experience of treating various diseases such as COVID-19 are crucial for designing fuzzy traffic controller in formulating linguistic protocols that generate the control input to the control system. A total of 3,888 (3 3 3 3 3 4 2 2) rules are formed based on eight input parameters and one output, which gives the risk level of COVID-19, five in number, to the diabetic patients. Risk level 1 is the lowest risk, while risk level 5 is the highest risk. With the help of various state-of-the-art machine learning techniques, fifteen models were built, namely logistic regression, AdaBoost, CatBoost, gradient boosting, random forest, extreme gradient boosting, extra trees, light gradient boosting machine, decision tree, linear discriminant analysis, K-neighbors, SVM-linear kernel, ridge, naive Bayes, and quadratic discriminant analysis. The performance of these fifteen models in terms of accuracy, recall, precision, F1 score, and kappa score has been calculated. The hyper-parameter approach further optimizes the best performer model. The block diagram of the proposed inference pipeline is shown in Figure 1.

The major contributions of the work are as follows:

- The impact of COVID-19 over diabetic patients is identified using a fuzzy inference system (FIS) and machine learning (ML) techniques.
- Various machine learning models are trained using various ML techniques, and the performance is validated through stratified K-fold cross-validation. Chances of bias and variance problems are neutralized.
- The output ML model can be directly used to validate the actual data and a learning metric to make the current model precise.

The remaining part of the study is carried out as follows. The fuzzy model for the proposed eight-input fuzzy traffic controller, fuzzy set membership functions for input and output variables, and the proposed work's rule base are all described in Section 2. Details of the simulation are given in Section 3.  Section 4 presents the machine learning models, along with results obtained from various machine learning models. Finally, Section 5 concludes the work with a brief discussion.

## 2. Fuzzy Inference System

A fuzzy logic-based controller is proposed for estimating the risk level of COVID-19 for the diabetic patients with eight input parameters, namely fever, cough, sore throat, cardiovascular disease, high blood pressure, age, sex, and travel history for the last three weeks and one output, which gives the risk level of COVID-19, five in number, to the diabetic patients. Risk level 1 is the lowest risk, while risk level 5 is the highest risk. Fuzzy sets of various levels of cough have been taken as low, medium, and high. Cough level from none to mild refers to low, from mild to moderate as medium, and moderate to severe as high. All five levels of cough, namely chest cough, dry tickling cough, bronchitis, post-viral cough, and whooping cough, have been considered [26].

Fuzzy sets of various levels of fever have been taken as low, medium, and high. Fever level from 98.0°F to 99°F refers to low, from 98.0°F to 101°F as medium, and 100.0°F and above as high. It covers all stages of fever such as no sign of fever, prodromal stage, second stage or chill, third stage, or flush or defervescence [27]. Fuzzy sets of various levels of the sore throat have been taken as low, medium, and high. No sign of cough to stage 1 of cough refers to low, stage 1 to stage 2 as a medium, and stage 2 to stage 3 as high. All three stages of the sore throat have been considered. The patient may feel exhausted, fatigued, and have a runny or congested nose in stage 1. The patient may suffer a runny nose, slight pains, sneezing, sleepiness, fatigue, or cough at this stage of the cold in stage 2. Stage 3 is the most severe stage of a cold during which the patient may experience congestion, a sore throat, and other symptoms [28].

Fuzzy sets of various levels of cardiovascular disease have been taken as low, medium, and high. No sign of cardiovascular disease to stage B of cardiovascular disease refers to low, stage A to stage C as a medium, and stage B to stage *E* as high. Stage A is thought of as a pre-heart collapse. Stage B can also be regarded as pre-heart failure diagnosed with systolic left ventricular dysfunction but has not had signs of heart failure. An echocardiogram (echo) that reveals that an ejection fraction (EF) of 40% or less and decreased EF (HFrEF) owing to specific causes are considered in stage B. Patients who have been recognized with heart disease and have (now) or had (previously) symptoms and indicators of the condition are regarded in stage C. In stage *D*, E patients who do not get better with therapy are considered [29].

Fuzzy sets of various high blood pressure levels have been low, medium, and high. High blood pressure from 110 to 120 refers to low, 115 to 135 as a medium, and 130 to 140+ as high [30]. The case fatality rate for COVID-19 is found to be nearly 1.4% with age. Here, 63% of coronavirus deaths in India have been observed in the 60+ age group as per the Health Ministry of the Government of India, which is in line with international data of COVID-19 fatality rates. Considering this, fuzzy sets of age have been considered low, medium, high, and very high. Age from 0 to 20 years refers to low, 15 to 35 years as a medium, 35 to 55 as high, and 45 and above as high.

Sex has also played an essential role in COVID-19. Data show that males have a significantly higher chance of having acute symptoms and dying than females. Data accumulated by Global Health 50/50 [31] were considered. In Italy, the number of death cases observed to be 71% male and 29% females, while Spain has observed 65% credited to males, with 35% constituting females.

A mean of all significant nations has been taken that gives 61.8% of case deaths caused to male with 38.2% being female. Considering these factors, fuzzy sets of sex have been taken as low and high. Gender female refers to low, while gender male refers to high. Fuzzy sets of travel history during the last 3 weeks have been taken as low and high. During the last 3 weeks, no travel history refers to low, while if so, then it is high (Table 1).

The proposed version has 3 subprocesses, i.e., fuzzification, fuzzy inference, and defuzzification. Throughout fuzzification, sharp values are converted into fuzzy sets supporting membership purposes. Afterwards, these fuzzy sets are passed into the rule base, i.e., if-then statements. Finally, fuzzy sets of the input and output factors are displayed in Table 2.

The final phase of this paradigm is defuzzification, which involves using the fuzzy rule basis to create crisp output signal values. It is the inverse of the fuzzification procedure. Mamdani devised a method of inference based on centroid defuzzification, which was used to turn fuzzy locations into crisp values. The membership functions are shown in Figure 2.

The rule base of the fuzzy set is shown in Table 3. A total of 3,888 (3^*∗*^3^*∗*^3^*∗*^3^*∗*^3^*∗*^4^*∗*^2^*∗*^2) rules are formed based on eight input parameters and one output, which gives the risk level of COVID-19, five in number, to the diabetic patients. Thus, risk level 1 is the lowest risk, while risk level 5 is the highest risk.

## 3. Simulation

The simulation was carried out with the help of MATLAB 8.1 and the fuzzy logic toolbox. For two reasons, the fuzzy logic toolbox was employed. To begin with, this toolbox may be used to quickly and easily create a rule basis, and updates can be made as needed. Second, it lowers the time it takes to construct the rule base. Table 3 demonstrates the rule base for various input variables and outcomes.  Table 4 shows a sample of eight outputs.

## 4. Machine Learning Models

It is categorised as a multiclass classification problem based on eight inputs and one output parameter, i.e., target variable. During the data preprocessing phase, the crisp values of input and output parameters are converted into numeric values. Once the dataset is ready, it is used to train and test using various machine learning models. Fifteen machine learning models are used for this purpose, namely logistic regression, AdaBoost, CatBoost, gradient boosting, random forest, extreme gradient boosting, extra trees, light gradient boosting machine, decision tree, linear discriminant analysis, K-neighbors, SVM-linear kernel, ridge, Naïve Bayes, and quadratic discriminant analysis. Furthermore, a few parameters have been chosen to calculate the performance of these fifteen models: accuracy, AUC, recall, precision, F1, and kappa scores. Based on the values of these parameters, the best model among these fifteen models is selected. Finally, hyper-parameter tuning is performed based on the dataset and various patterns for better performance.

Performance characteristics of ML techniques on COVID-19 symptoms are shown in Table 1. Five performance characteristics are used: accuracy, recall, precision, F1 score, and kappa score. Except for F1 score, all parameters are independently derived, whereas F1 score is derived using recall and precision. Except for the AUC score, all parameter follows the same trend. It is observed that the logistic regression model gives the best performance, followed by the AdaBoost and CatBoost classifier. These characteristics can further be improved using the hyper-parameter optimization process.

The performance metrics that were used in this work are accuracy, recall, precision, F1 score, kappa, confusion matrix, ROC, and AUC curves. Additionally, learning rate graphs were also drawn alongside the number of training instances. Accuracy purely defines the chances of identifying the correct class from all other classes. Precision is the ratio of correctly classifying the class, positive classifications from all the positive classifications. Higher precision means fewer chances of misclassifying a class as not that particular class. At the same time, recall or sensitivity helps to identify and revisit the observations that were correctly classified from all the possible true observations in the experiment. F1 score is the weighted average of both precision and recall, which can help to identify the uneven class distribution. In this case, the classes are evenly distributed. Therefore, it is not preferred over accuracy. Hence, only accuracy scores are discussed widely. Similarly, kappa values describe the distribution of the class variable and data collection. Since the current dataset is created from a fuzzy rule base, this metric does not add any value over accuracy. Table 1 represents each machine learning model and its respective performance parameters such as accuracy, recall, precision, F1 score, and kappa score. Based on these scores, one would pick the appropriate models, preferably testing and predicting further use cases. However, since these models are not perfect, they can be further used by tuning the algorithm's hyper-parameters while training the model. After this process, bar graphs are drawn for each model and each of their performance metric (Figures 3–7). Observing these findings, CatBoost, logistic regression, and XGBoost improved their performance. Every model created from these algorithms showed significant improvement, followed by hyper-parameter optimization. CatBoost showed almost a 3% improvement in its accuracy. Logistic regression and XGBoost got improved over 1.1% and 3%, respectively. Each model is now executed for various performance attributes of accuracy, recall, precision, F1 score, and kappa score. Hyper-parameter optimization is used to improve performance further. The accuracy, recall, precision, F1 score, and kappa score after hyper-parameter optimization are shown in Figures 3-7 respectively.

The CatBoost classifier gives the highest accuracy, recall, precision, F1 score, and kappa score.

The CatBoost classifier model is selected for testing over the confusion matrix. Figures 8-9 show the confusion matrices of CatBoost classifier before and after hyper-parameter tuning. ROC curve is drawn against false-positive rate and accurate positive rate prediction scores of the CatBoost model after hyper-parameter optimization, which tells whether the model is going wrong. For all five classes of the output parameter, AUC scores were observed as substantially good, approaching 1.  Figure 10 shows the ROC curve for the CatBoost classifier with AUC scores. After hyper-parameter optimization, this CatBoost classifier model is trained and tested again for about 2500 instances. Again, stratified k-fold cross-validation is used, which reaches about 74% accuracy. The shaded area around the line is the variance of accuracy.  Figure 11 shows the validation of training and cross-validation scores. As the current model is a multinomial decision-making problem, a set of these classifications, decision-making, and ensemble algorithms is used in Figure 8. Specific performance parameters are used to validate the model, such as AUC and confusion matrix. The area under the curve (AUC) is generally used to validate the model's performance. AUC is decided using measures such as true-positive rate (TPR) and false-positive rate (FPR). A confusion matrix is a good measure to identify true positives, true negatives, false positives, and false negatives using TPR and FPR calculated. If the FPR is higher, the graph generally tends to drop below the region of operation (which is a diagonal line from the origin), making the model unusable. As a rule of thumb, the AUC score should generally be more than 0.5, above the diagonal line. On the other hand, the TPR would be higher if the model finds the best fit. In such a case, CatBoost is observed to have better TPR since most of the data are categorical.

Table 5 shows the top three best performing models after tuning hyper-parameter in accuracy, recall, precision, F1 score, and kappa score.

While modelling a machine learning model, one could come across the term hyper-parameters. Hyper-parameters are not updated while training the model, whereas the model is trained over an algorithm and validated based on its accuracy. Therefore, these hyper-parameters welcome new possibilities to improve the existing machine learning model. Though many other parameters can explain the model performance such as accuracy, recall, precision, F1 score, kappa score, and AUC, modelling the accuracy is only considered. Therefore, hyper-parameters help to improve performance. Hyper-parameter optimization maintains the existing accuracy and improves other parameters that enhance the overall performance of the machine learning model. This can be achieved by employing an optimization problem on top of the existing model, searching for the best hyper-parameter. A randomized grid search is opted to explore the appropriate parameters to improve AUC and accuracy scores for the current scenario. CatBoost classifier is the current state-of-the-art performer for decision-making using gradient boosting algorithms. It is an ensemble technique such as extra trees, AdaBoost, and XGBoost classifier, but it comes with way better parametric identification as it demands categorical features in case of any. The entire dataset combines categorical values, both input and output in the current work. Therefore, the problem is fitted to the exact use case for CatBoost after grid searching the major hyper-parameters such as learning rate (0.05) and depth (6). Other hyper-parameters were either machine-specific or data-specific, and hence, they were set to their defaults. After implementing the algorithm with the updated hyper-parameters, the model's performance was the best among the other algorithms. Generally, the logistic regression algorithm is preferred for binary classification. For logistic regression classifiers, the hyper-parameters are solver, penalty, C, and max iterations. These parameters play a crucial role in the performance of the model. For this work, Sklearn offers five options for solver and saga (stochastic average gradient descent with L1 regularisation). C is the strength of the penalty, which is identified to be 7.0028. Since the data are not massive, the maximum number of iterations was set to default. XGBoost is a gradient boosting technique in the decision-making process, which also comes with a few hyper-parameters, and after grid searching, the following are discovered: min child weight = 7, max depth = 6, learning rate = 0.1, gamma = 0.4, and sample tree = 0.5. There are other parameters in XGBoost, but these parameters affected AUC and accuracy the most.

## 5. Conclusion

Although diabetes was associated with worse results in COVID-19 patients, no clinical report demonstrates the susceptibility concerning COVID-19 to be greater in people with diabetes. In a few recent findings, it is found that humans are twice as likely to die from complications of diabetes. The overall mortality of COVID-19 in China from January to April 2020 was almost thrice higher in patients with diabetes. Given the multifold mortality rate of COVID-19 in diabetic patients, this work proposes the COVID-19 risk prediction model for diabetic patients using a fuzzy inference system and machine learning approaches to estimate the risk level of COVID-19 in diabetic patients, making it possible for timely action. The proposed model also helps minimise the medical practitioner's advice for estimating the risk level of COVID-19 for diabetic patients, which is mainly engaged in treating COVID-19 patients. The proposed model takes eight input parameters that were found as the most influential symptoms in diabetic patients who contracted COVID-19, namely fever, cough, sore throat, cardiovascular disease, high blood pressure, age, sex, and travel history for the last three weeks. A total of 3,888 (3^*∗*^3^*∗*^3^*∗*^3^*∗*^3^*∗*^4^*∗*^2^*∗*^2) rules were formed based on eight input parameters and one output, which gives the risk level of COVID-19 for diabetic patients, five in number, to the diabetic patients. Risk level 1 is the lowest, while level 5 is the highest. With the help of various state-of-the-art machine learning techniques, fifteen models were built, namely logistic regression, AdaBoost, CatBoost, gradient boosting, random forest, extreme gradient boosting, extra trees, light gradient boosting machine, decision tree, linear discriminant analysis, K-neighbors, SVM-linear kernel, ridge, naïve Bayes, and quadratic discriminant analysis. The CatBoost classifier gives the best accuracy, recall, precision, F1 score, and kappa score. After hyper-parameter optimization, the CatBoost classifier showed 76% accuracy and improvements in the recall, precision, F1 score, and kappa score, followed by logistic regression and XGBoost with 75.1% and 74.7% accuracy. Stratified k-fold cross-validation was used for validation purposes. Though the fuzzy inference system's knowledge base provides reasonably good insights, accuracy and precision can be improved with the actual medical record. A better synthetic data generation technique can eliminate the slight bias of being completely naive and variance fluctuations, avoiding hyper-parameter optimization.

## Figures and Tables

**Figure 1:** Proposed inference pipeline.

**Figure 2:** Fuzzy set membership diagrams.

**Figure 3:** Comparison of accuracy after hyper-parameter optimization.

**Figure 4:** Comparison of recall after hyper-parameter optimization.

**Figure 5:** Comparison of precision after hyper-parameter optimization.

**Figure 6:** Comparison of kappa score after hyper-parameter optimization.

**Figure 7:** Comparison of F1 score after hyper-parameter optimization.

**Figure 8:** Confusion matrices of CatBoost classifier before hyper-parameter tuning.

**Figure 9:** Confusion matrices of CatBoost classifier after hyper-parameter tuning.

**Figure 10:** ROC curve for CatBoost classifier with AUC scores.

**Figure 11:** Validation of training and cross-validation scores.

**Table 1:** Performance characteristics of ML techniques on COVID-19 symptoms.

S. no	Model	Accuracy	Recall	Precision	F1 score	Kappa
1	Logistic regression	0.7391	0.503	0.7536	0.7195	0.5995
2	AdaBoost classifier	0.7324	0.549	0.7433	0.7093	0.5908
3	CatBoost classifier	0.7166	0.601	0.7159	0.7136	0.5817
4	Light gradient boosting machine	0.7041	0.557	0.7031	0.6997	0.561
5	Gradient boosting classifier	0.6968	0.483	0.7052	0.6816	0.537
6	Extreme gradient boosting	0.6935	0.473	0.7037	0.6757	0.5303
7	Extra trees classifier	0.6928	0.562	0.6929	0.6908	0.5494
8	Decision tree classifier	0.6909	0.59	0.697	0.6922	0.5501
9	Random forest classifier	0.6909	0.558	0.6898	0.6884	0.5459
10	SVM-linear kernel	0.6733	0.449	0.703	0.639	0.4971
11	K-neighbor classifier	0.6534	0.495	0.6474	0.6461	0.485
12	Ridge classifier	0.6487	0.345	0.4885	0.5572	0.4365
13	Quadratic discriminant analysis	0.5182	0.426	0.5352	0.5067	0.3164
14	Naive Bayes	0.4943	0.493	0.6474	0.5279	0.3152

**Table 2:** Input/output variables and their fuzzy sets.

Input/output variables	Fuzzy sets
Cough (Input 1)	*{*Low, medium, high*}*
Fever (Input 2)	*{*Low, medium, high*}*
Sore throat (Input 3)	*{*Low, medium, high*}*
Cardiovascular disease (Input 4)	*{*Low, medium, high*}*
High blood pressure (Input 5)	*{*Low, medium, high*}*
Age (Input 6)	*{*Low, medium, high, very high*}*
Sex (Input 7)	*{*Low, high*}*
Travel history during the last 3 weeks (Input 8)	*{*Low, high*}*
Prescription (output)	*{*Risk level 1, 2, 3, 4, 5*}*

**Table 3:** Rule base of the fuzzy inference.

Sl. no.	Input parameters								Output parameter
	Cough	Fever	Sore throat	Cardio. Disease	B.P.	Age	Sex	Travel history	Risk level
1	Low	Low	Low	Low	Low	Low	Low	Low	Risk level 1
2	Medium	Low	Low	Low	Low	Low	Low	Low	Risk level 1
3	High	Low	Low	Low	Low	Low	Low	Low	Risk level 1
4	Low	Medium	Low	Low	Low	Low	Low	Low	Risk level 1
5	Medium	Medium	Low	Low	Low	Low	Low	Low	Risk level 1
6	High	Medium	Low	Low	Low	Low	Low	Low	Risk level 1
7	Low	High	Low	Low	Low	Low	Low	Low	Risk level 1
8	Medium	High	Low	Low	Low	Low	Low	Low	Risk level 1
9	High	High	Low	Low	Low	Low	Low	Low	Risk level 1
10	Low	Low	Medium	Low	Low	Low	Low	Low	Risk level 1
. . .	. . .	. . .	. . .	. . .	. . .	. . .	. . .	. . .	. . .
. . .	. . .	. . .	. . .	. . .	. . .	. . .	. . .	. . .	. . .
. . .	. . .	. . .	. . .	. . .	. . .	. . .	. . .	. . .	. . .
3888	High	High	High	High	High	Very high	High	High	Risk level 5

**Table 4:** Sample of eight outputs.

Cough	Fever	Sore throat	Cardiovascular disease	BP	Age	Sex	Travel history	Prescription
3	101.5	0.5	4.5	120	27	0.5	0.5	Risk level 2
2	105	0.6	5	110	37.5	0.8	0.8	Risk level 3
5	103	0.3	4	140	47	0.6	0.8	Risk level 4
5	105	0.8	5	150	32	0.4	0.7	Risk level 5
2	99	0.3	4	110	48	0.5	0.4	Risk level 1
6	99	0.6	3	120	25	0.4	0.4	Risk level 2
6	103	0.2	6	125	20	0.5	0.8	Risk level 4
2	98	0.6	5	135	55	0.3	0.3	Risk level 3

**Table 5:** Top three best performing models after tuning hyper-parameter.

S. no.	Model	Accuracy	Recall	Precision	F1 score	Kappa score
1	CatBoost classifier	0.7582	0.64	0.772	0.767	0.663
2	Logistic regression	0.751	0.57	0.753	0.731	0.631
3	XGBoost classifier	0.7471	0.55	0.727	0.721	0.591

## Data Availability

No data were used to support this study.
